# microRNA-526b servers as a prognostic factor and exhibits tumor suppressive property by targeting Sirtuin 7 in hepatocellular carcinoma

This article has been retracted.

**DOI:** 10.18632/oncotarget.21209

**Published:** 2017-09-23

**Authors:** Xin Liu, Liu Yang, Jianfeng Tu, Wenwei Cai, Meiqi Zhang, Zhangxuan Shou, Yingmin Yao, Qiuran Xu

**Affiliations:** ^1^ Key Laboratory of Tumor Molecular Diagnosis and Individualized Medicine of Zhejiang Province, Zhejiang Provincial People's Hospital, People's Hospital of Hangzhou Medical College, Hangzhou, Zhejiang Province 310014, China; ^2^ Department of Emergency, Zhejiang Provincial People's Hospital, People's Hospital of Hangzhou Medical College, Hangzhou, Zhejiang Province 310014, China; ^3^ Department of Pharmacy, Zhejiang Provincial People's Hospital, People's Hospital of Hangzhou Medical College, Hangzhou, Zhejiang Province 310014, China; ^4^ Department of Hepatobiliary Surgery, The First Affiliated Hospital of Xi'an Jiaotong University, Xi'an, Shaanxi Province 710061, China

**Keywords:** miR-526b, HCC, tumor growth, metastasis, SIRT7

## Abstract

Recent studies have reported that microRNA-526b (miR-526b) is implicated in the growth and metastasis of cancer cells. However, the clinical significance of miR-526b and its role as well as underlying mechanisms are largely unknown in hepatocellular carcinoma (HCC). Here, we detected miR-526b expression difference between HCC and matched nontumor tissues with qRT-PCR. We found that miR-526b displayed lower expression in HCC patient tissues and cells. Clinical analysis revealed that low miR-526b expression correlated with large tumor size, venous infiltration, advanced tumor-node-metastasis (TNM) stage. Furthermore, miR-526b underexpression independently predicted poor prognosis of HCC patients. Functionally, we demonstrated that miR-526b inhibited proliferation, migration and invasion of HCC cells *in vitro*. Moreover, miR-526b overexpression restrained the tumor growth and pulmonary metastasis *in vivo*. Mechanistically, we proved that miR-526b could directly bind to 3′UTR of sirtuin 7 (SIRT7) mRNA and repressed its expression. miR-526b and SIRT7 showed a negative correlation in HCC tissues. More importantly, up-regulating SIRT7 expression antagonized miR-526b-inhibited proliferation, migration and invasion in SMMC-7721 cells. Furthermore, miR-526b suppressed epithelial-to-mesenchymal transition (EMT) of HCC cells. Immunoblotting analysis indicated that miR-526b reduced the levels of phosphorylated ERK (p-ERK), c-Myc, Cyclin D1, c-Jun, SNAIL and SLUG in HCC cells. SIRT7 restoration promoted phosphorylation of ERK and EMT in miR-526b overexpressing SMMC-7721 cells. Taken together, this is the first time we demonstrated that miR-526b might function as a prognostic biomarker and suppressed SIRT7 expression, and subsequently led to the growth and metastasis of HCC. Our findings provide miR-526b/SIRT7 axis as a promising drug target for HCC.

## INTRODUCTION

Hepatocellular carcinoma (HCC) is one of the most common malignancies and a highly invasive tumor with frequent distant metastasis in China [1, 2]. Its incidence has increased in recent years, but it has not yet achieved satisfactory curative effect [1]. Therefore, it is important to elucidate the precise molecular mechanisms of HCC development and develop new therapeutic targets [3].

MicroRNAs (miRNAs) regulate gene expression via the degradation of mRNA or inhibition of translation. Numerous studies have demonstrated that miRNAs play essential roles in regulating initiation and progression of HCC [4–6]. miR-526b is identified as a pregnancy-associated miRNAs and locates on chromosome 19q13.42 [7–10]. miR-526b suppresses the transcriptional activity of lincRNA-NR_024015 by directly binding and inhibits cell proliferation in non-cardia gastric cancer [11]. The G to A base change at miR-526b binding-site in the lincRNA-NR_024015 exon resistances to transcriptional inhibition of miR-526b and associates with poor clinical outcome of esophageal squamous cell carcinoma (ESCC) [12]. miR-526b underexpression predicts poor prognosis of non-small cell lung cancer (NSCLC) patients and prohibits the growth of NSCLC cells *in vitro* and *in vivo* by targeting Ku80 [13]. Matrix metalloproteinase 1 (MMP1) is recognized as a direct target of miR-526b in dermal fibroblasts [14]. Furthermore, miR-526b-3p exhibits tumor suppressive property by suppressing glycolysis, metastasis and proliferation of colon cancer cells, and hypoxia-inducible factor 1-alpha (HIF-1α) functions as a critical mediator of miR-526b-3p [15]. Notably, miR-526b is up-regulated COX-2 and enhances tumorsphere formation, epithelial-to-mesenchymal transition (EMT), invasion, migration of breast cancer cells [16]. These published studies show that the expression and role of miR-526b is a controversial topic in human cancer. To date, the expression and role of miR-526b is rarely investigated in HCC.

In this study, aberrant upregulation of miR-526b expression was detected in HCC tissues. miR-526b overexpression associated with poorer prognostic features and shorter survival of HCC patients. We presented evidence that miR-526b inhibited proliferation, metastasis and EMT of HCC cells by targeting sirtuin 7 (SIRT7). Our results reveal a novel molecular mechanism that miR-526b/SIRT7 axis may be a valuable clinical marker and therapeutical target for HCC patients.

## RESULTS

### miR-526b expression is down-regulated in HCC

The expression differences of miR-526b between 80 HCCs and matched tumor-adjacent tissues were investigated. The qRT-PCR analysis revealed that miR-526b expression was markedly decreased in HCC tissues compared with adjacent noncancerous tissues (P<0.05, Figure 1A). In accordance, we found that the miR-526b level was significantly down-regulated in HCC cell lines (HepG2, Hep3B, SMMC-7721 and Huh7) compared with normal hepatic cell line LO2 (P<0.05, respectively, Figure 1B). The findings provide valid evidence that miR-526b may be implicated in pathogenesis and development of HCC.

**Figure 1:** Aberrant expression and prognostic significance of miR-526b in HCC **(A)** Eighty paired of HCC and tumor-adjacent tissues were subjected to qRT-PCR for miR-526b expression. Quantitative data revealed that miR-526b expression was decreased in HCC tissue compared with tumor-adjacent tissues. ^*^P<0.05 by t test. **(B)** The differences in the expression of miR-526b between four different HCC cells lines (Hep3B, HepG2, SMMC-7721 and Huh7) and the human immortalized normal hepatic cell line (LO2). n = three repeats with similar results, ^*^P<0.05 by ANOVA, respectively. **(C)** Different subgroups (miR-526b low/high expression) were plotted according to the cutoff values of miR-196b, which were defined as the median of the cohort. HCC patients whit low miR-526b level showed a significant shorter overall survival. P<0.05 by Log-rant test.

### miR-526b expression correlates with the prognosis of HCC patients

Different subgroups (miR-526b low/high expression) were plotted according to the cutoff values of miR-526b, which were defined as the median of the cohort. Relationship between clinical characteristics of the HCC patients and miR-526b expression were listed in Table 1. Low miR-526b expression was associated with large tumor size (P=0.022), venous infiltration (P=0.014) and advanced tumor-node-metastasis (TNM) tumor stage (P=0.045). Furthermore, survival analyses indicated that HCC patients with low miR-526b level showed a significant shorter 3-year overall survival (P=0.041, Figure 1C). Multivariate Cox regression analysis revealed that miR-526b underexpression independently predicts poor prognosis of HCC patients (P=0.021, Table 2). Thus, we suggest that miR-526b is a promising prognostic biomarker for HCC patients.

**Table 1:** Clinicopathological correlation analysis of miR-526b expression in hepatocellular carcinoma

Clinicopathologic features		miR-526b expression		*P*
		High level (n=40)	Low level (n=40)	
Age (y)	≤50	15	17	0.648
	>50	25	23	
Sex	Male	33	35	0.531
	Female	7	5	
HBsAg	No	4	7	0.330
	Yes	36	33	
Serum AFP level (ng/mL)	≤20	14	10	0.329
	>20	26	30	
Tumor size (cm)	≤5	15	6	0.022^*^
	>5	25	34	
No. of tumor nodules	1	36	32	0.210
	≥2	4	8	
Cirrhosis	Absent	13	7	0.121
	Present	27	33	
Venous infiltration	Absent	25	14	0.014^*^
	Present	15	26	
Edmondson-Steiner grading	I+II	34	27	0.066
	III+IV	6	13	
TNM tumor stage	I+II	36	29	0.045^*^
	III+IV	4	11	

HBV, hepatitis B virus; AFP, alpha-fetoprotein; TNM, tumor-node-metastasis. ^*^Statistically significant.

**Table 2:** Multivariate Cox regression analysis of overall survival in hepatocellular carcinoma patients

Variables	OS		
	HR	95% CI	*P*
No. of tumor nodules	2.114	1.113-3.815	0.044^*^
Tumor size	2.231	1.109-4.275	0.032^*^
Venous infiltration	2.327	1.206-4.712	0.019^*^
Edmondson-Steiner grading	1.814	1.121-2.973	0.041^*^
TNM tumor stage	2.362	1.157-4.213	0.026^*^
miR-526b expression	0.255	0.082-0.076	0.021^*^

TNM, tumor-node-metastasis; HR, hazard ratio; CI, confidence interval. ^*^Statistically significant.

### miR-526b suppresses proliferation, migration and invasion of HCC cells

To detect the effects of miR-526b on proliferation, migration and invasion of HCC cells, CCK-8 proliferation assay and Transwell assay were conducted when miR-526b expression was down-regulated or up-regulated in HCC cells. miR-526b was obviously up-regulated by miR-526b mimic in SMMC-7721 cells (P<0.05, Figure 2A). CCK-8 assays indicated that miR-526b restoration notably restrained the proliferation of SMMC-7721 cells (P<0.05, Figure 2B). Transwell assays revealed that miR-526b overexpression significantly weakened the migratory and invasive abilities of SMMC-7721 cells (P<0.05, respectively, Figure 2C). In accordance, miR-526b knockdown was confirmed by qRT-PCR after miR-526b inhibitor transfection in Hep3B cells (P<0.05, Figure 2D). Our data showed that down-regulating miR-526b expression significantly enhanced proliferation, migration and invasion of Hep3B cells compared with control groups (P<0.05, respectively, Figure 2E and 2F). Building on these findings *in vitro*, we further probed the role of miR-526b during HCC progression with xenograft models. Notably, ectopic expression of miR-526b resulted in a notable decrease of tumor growth and reduced metastasis nodes in lung compared with control groups (P<0.05, respectively, Figure 3A and 3B). Thus, miR-526b exerts a tumor suppressive role in HCC.

**Figure 2:** miR-526b inhibits proliferation, migration and invasion of HCC cells **(A)** SMMC-7721 cells that were transfected with miR-526b mimic or negative control (NC) mimic were detected by qRT-PCR for miR-526b expression. n = three repeats with similar results, ^*^P<0.05 by t test. **(B)** CCK-8 assays revealed that miR-526b silencing inhibited proliferation of SMMC-7721 cells. n = three repeats with similar results, ^*^P<0.05 by ANOVA. **(C)** Transwell assays confirmed that miR-526b overexpression restrained migration and invasion of SMMC-7721 cells. n = three repeats with similar results, ^*^P<0.05 by t test, respectively. **(D)** Hep3B cells were transfected with miR-526b inhibitor and negative control (NC) inhibitor, respectively, and measured by qRT-PCR for miR-526b expression. n = three repeats with similar results, ^*^P<0.05 by t test. **(E)** and **(F)** upregulating miR-526b expression enhances proliferative, migratory and invasive abilities of Hep3B cells. n = three repeats with similar results, ^*^P<0.05 by ANOVA and t test, respectively.

**Figure 3:** miR-526b restoration restrains tumor growth and lung metastasis of HCC in mice **(A)** SMMC-7721 cells that were transfected with miR-526b mimic or negative control (NC) mimic were subcutaneously injected into the flank of nude mice. Tumor growth curves indicated that miR-526b overexpression prohibited the growth of SMMC-7721 cells *in vivo*. n = 6, ^*^P<0.05 by t test. Scale bar: 1 cm. **(B)** miR-526b overexpressing SMMC-7721 cells were intravenously injected into nude mice via tail vein. Lungs of mice were sectioned and stained by H&E. miR-526b overexpression significantly reduced the number of metastatic nodules in mice lungs. n = 6, ^*^P<0.05 by t test.

### miR-526b directly targets SIRT7 in HCC

In order to explore the molecular mechanisms underlying miR-526b, first, bioinformatic prediction (TargetScan: http://www.targetscan.org and miRanda: http://www.microrna.org/microrna/hpme.do) showed that miR-526b could bind to 3′UTR of SIRT7 mRNA (Figure 4A). qRT-PCR and immunoblotting results indicated that miR-526b overexpression reduced the levels of SIRT7 mRNA and protein in SMMC-7721 cells (P<0.05, respectively, Figure 4B). miR-526b silencing increased the expression of SIRT7 in Hep3B cells (P<0.05, respectively, Figure 4C). To further confirm the binding of miR-526b and 3′UTR of SIRT7, a dual-luciferase reporter assay was implemented. Co-transfection of Hep3B cells with Pmir-RB-SIRT7 vector and miR-526b mimic or inhibitor significantly modulated luciferase reporter activity compared with the negative control (P<0.05, respectively, Figure 4D). These regulatory effects were abolished by directed mutagenesis of the miR-526b binding seed region in 3′UTR of SIRT7 (Figure 4D). Recent study found that SIRT7 was prominently overexpressed in HCC tissues and showed an oncogenic potential [17, 18]. The data from qRT-PCR demonstrated that the expression of SIRT7 mRNA in HCC tissues was notably up-regulated compared to normal liver tissues (P<0.05, Figure 5A). Moreover, IHC data revealed that 13 of 20 (65.0%) HCC tissues showed positive expression of SIRT7, while SIRT7 positive staining was only detected in 5 of 20 (25.0%) tumor-adjacent tissues (P<0.05, Figure 5B). Subsequently, a significant negative correlation between miR-526b and SIRT7 expression was observed in HCC tissues (r=-0.708, P<0.001, Figure 5C). Different subgroups (SIRT7 low/high expression) were plotted according to the cutoff values of SIRT7, which were defined as the median of the cohort. HCC patients with high SIRT7 level showed large tumor size (P=0.005, Supplementary Table 1), venous infiltration (P=0.044, Supplementary Table 1) and advanced TNM stage (P=0.002, Supplementary Table 1). Otherwise, western blotting was performed to detect the levels of HIF1α, MMP1 and Ku80, which were identified as direct targets of miR-526b [13–15]. miR-526b restoration did not affect the levels of HIF1α, MMP1 and Ku80 in SMMC-7721 cells (Supplementary Figure 1). Together, these data demonstrate that SIRT7 is a direct target of miR-526b in HCC.

**Figure 4:** SIRT7 is a direct target of miR-526b in HCC **(A)** The sequences of wild type (wt) or mutant (mt) SIRT7-3′UTR were cloned into the pmiR-RB-Report™ vector. **(B)** SMMC-7721 cells were transfected with miR-526b mimic or negative control NC) mimic and measured by qRT-PCR and immunoblotting for SIRT7. n = three repeats with similar results, ^*^P<0.05 by t test. **(C)** miR-526b knockdown increased the level of SIRT7 in Hep3B cells. n = three repeats with similar results, ^*^P<0.05 by t test. **(D)** Co-transfection of Hep3B cells with Pmir-RB-SIRT7 vector and miR-526b mimic or inhibitor significantly modulated luciferase reporter activity compared with the negative control. miR-526b mimic or inhibitor showed no significant effect on luciferase reporter activity of mt SIRT7-3′UTR. n = three repeats with similar results, ^*^P<0.05 by t test.

**Figure 5:** miR-526b inversely correlated with SIRT7 in HCC **(A)** The data from qRT-PCR analysis confirmed the up-regulation of SIRT7 in HCC tissues. ^*^P<0.05 by t test. **(B)** Representative IHC staining indicated that strong staining of SIRT7 was observed in HCC tissues, while matched tumor-adjacent tissues showed weak signal of SIRT7. Scale bar: 50μm. **(C)** An obvious negative correlation between miR-526b and SIRT7 expression was observed in HCC tissues. n = 80, P<0.05 by Pearson's correlation analysis.

### SIRT7 functions in miR-526b-regulated proliferation, migration and invasion of HCC cells

Next, we tested whether SIRT7 was able to mediate the function of miR-526b in HCC cells. Co-transfection of miR-526 mimic+SIRT7 vector could rescue the miR-526b-induced downregulated expression of SIRT7 in SMMC-7721 cells (P<0.05, Figure 6A). Furthermore, SIRT7 restoration enhanced the proliferation of SMMC-7721 cells with miR-526b overexpression (P<0.05, Figure 6B). In accordance, Forced expression of SIRT7 promoted the migration and invasion of miR-526b overexpressing SMMC-7721 cells (P<0.05. respectively, Figure 6C). Therefore, these results indicate that SIRT7 may function as a downstream mediator of miR-526b in HCC.

**Figure 6:** SIRT7 re-expression abrogates the effects of miR-526b in SMMC-7721 cells **(A)** SMMC-7721 cells that were underwent negative control (NC) mimic + empty vector (EV), miR-526b mimic + EV or miR-526b mimic + SIRT7 vector transfection were subjected to immunoblotting for SIRT7. n = three repeats with similar results, ^*^P<0.05 by ANOVA. **(B)** SIRT7 restoration enhanced proliferation of miR-526b overexpressing SMMC-7721 cells. n = three repeats with similar results, ^*^P<0.05 by ANOVA. **(C)** Re-expression of SIRT7 rescued the anti-cancer effects of miR-526b in SMMC-7721 cells. n = three repeats with similar results, ^*^P<0.05 by ANOVA.

### miR-526b inhibits HCC progression possibly by blocking ERK pathway

EMT has been recognized as a critical characteristic of invasive HCC [4]. Thus, we next detected the regulatory effects of miR-526b on EMT of HCC cells. Interestingly, miR-526b restoration significantly increased E-cadherin expression and reduced the level of Vimentin in SMMC-7721 cells (P<0.05, respectively, Figure 7A). In accordance, the morphology of miR-526 overexpressing SMMC-7721 cells showed more epithelial cell characteristics compared to control cells (Figure 7B). Moreover, miR-526b knockdown promoted the EMT of Hep3B cells (P<0.05, respectively, Figure 7C and 7D).

**Figure 7:** miR-526b prohibits EMT of HCC cells **(A)** SMMC-7721 cells that were transfected with miR-526b mimic or negative control (NC) mimic were detected by immunoblotting for E-cadherin and Vimentin. n = three repeats with similar results, ^*^P<0.05 by t test. **(B)** miR-526b overexpression resulted in MET of SMMC-7721 cells. **(C)** Hep3B cells were transfected with miR-526b inhibitor and negative control (NC) inhibitor, respectively, and measured by western blotting for E-cadherin and Vimentin. n = three repeats with similar results, ^*^P<0.05 by t test. **(D)** miR-526b knockdown promoted EMT of Hep3B cells.

Recent study reported that SIRT7 promoted growth, metastasis and EMT of colorectal cancer cells by activating Raf/MEK/ERK pathway [19]. Next, we checked whether miR-526b modulated ERK pathway by targeting SIRT7 in HCC cells. Notably, miR-526b overexpression obviously reduced the level of p-ERK without affecting total ERK expression in SMMC-7721 cells (P<0.05, respectively, Figure 8). And miR-526b overexpression accordingly decreased the levels of c-Myc, Cyclin D1, c-Jun, SNAIL and SLUG (P<0.05, respectively, Figure 8), which were downstream targets of ERK pathway. Meanwhile, miR-526b knockdown promoted the activation of ERK pathway in Hep3B cells (P<0.05, respectively, Figure 8). Moreover, re-expression of SIRT7 significantly increased the levels of p-ERK and Vimentin, and reduced E-cadherin expression in miR-526b overexpressing SMMC-7721 cells (P<0.05, respectively, Figure 9). Altogether, miR-526b prohibits proliferation, mobility and EMT of HCC cells possibly via inactivation of ERK pathway.

**Figure 8:** miR-526b inversely modulates ERK pathway in HCC cells SMMC-7721 cells that were transfected with miR-526b mimic or negative control (NC) mimic were detected by immunoblotting for p-ERK, ERK, c-Myc, Cyclin D1, c-Jun, SNAIL and SLUG. Hep3B cells were transfected with miR-526b inhibitor and negative control (NC) inhibitor, respectively. miR-526b knockdown increased the levels of p-ERK, ERK, c-Myc, Cyclin D1, c-Jun, SNAIL and SLUG in Hep3B cells. n = three repeats with similar results, ^*^P<0.05 by t test.

**Figure 9:** SIRT7 restoration reversed miR-526b-induced downregulation of p-ERK and MET in SMMC-7721 cells miR-526b overexpressingSMMC-7721 cells that were transfected with SIRT7 vector or empty vector (EV) were detected by immunoblotting for p-ERK, E-cadherin and Vimentin. Re-expression of SIRT7 significantly increased the levels of p-ERK and Vimentin, and reduced E-cadherin expression in miR-526b overexpressing SMMC-7721 cells. n = three repeats with similar results, ^*^P<0.05 by t test.

## DISCUSSION

Recently, more and more evidences have showed that miRNAs play a crucial role in tumorigenesis and development of tumor [20–22]. Searching a miRNA signature might be of clinical value for diagnosis, therapy and prognosis of HCC [22]. Aberrant expression of miR-526b has been reported in breast cancer [16], NSCLC [13] and colon cancer [15]. The prognostic significance of miR-526b was confirmed in breast cancer [16] and colon cancer [15]. Currently, the clinical significance of miR-526b was disclosed in HCC. We found that overexpression of miR-526b was associated with large tumor sized, venous infiltration and advanced TNM tumor stage. More importantly, low miR-526b level was independently predicts a significant shorter 3-year overall survival of HCC patients. Therefore, miR-526b potentially serves as a promising biomarker for the prognosis of HCC patients.

Tumor growth and metastasis are the root of poor clinical outcome for HCC patients [23]. Thus, investigating molecular mechanism involved in the proliferation, migration and invasion of HCC cells is beneficial to explore anti-cancer therapy. miR-526b is previously reported to regulate proliferation, migration and invasion of breast cancer and colon cancer [15, 16]. Thus, it is worth to disclose the role of miR-526b in HCC. Subsequently, our data showed that miR-526b inhibited proliferation, migration and invasion of HCC cells, and reduced tumor growth and lung metastasis in nude mice. Accordingly, we suggest that miR-526b exhibits tumor suppressive property in HCC. Bioinformatics analysis and subsequent experiments revealed that miR-526b directly targeted SIRT7 in HCC. SIRT7 is a newly identified oncogene or tumor suppressor, which exhibits an essential role in a wide range of biological processes including proliferation, cell cycle, chromatin regulation, chemotherapy resistance, cellular transformation and stress response [24]. SIRT7 exhibits an oncogenic role by promoting proliferation and cell cycle progression *in vitro* and facilitating *in vivo* growth of HCC [25]. Furthermore, miR-125a-5p and miR-125b are recognized as down-regulators of SIRT7 in HCC and bladder cancer [25, 26]. Rescue experiments indicated that SIRT7 was not only a downstream target but also a function mediator of miR-526b in HCC. Recent study reported that SIRT7 promoted growth, metastasis and EMT of colorectal cancer cells by activating Raf/MEK/ERK pathway [19]. Next, we demonstrated that miR-526b inhibited EMT of HCC cells. Western blotting analysis revealed that miR-526b led to inactivation of ERK pathway, which played an essential role in promoting HCC growth and metastasis [27]. It is reported that ERK could up-regulate c-Myc, Cyclin D1, c-Jun, SNAIL and SLUG expression [28–31]. Immunoblotting results found that expressions of c-Myc, Cyclin D1, c-Jun, SNAIL and SLUG were down-regulated in miR-526b-transfected cells. Furthermore, SIRT7 restoration reversed miR-526b-induced downregulation of p-ERK and MET in SMMC-7721 cells. Thus, miR-526b prohibits proliferation, mobility and EMT of HCC cells possibly via inactivation of ERK pathway.

In summary, analysis of HCC samples showed decreased levels of miR-526b that correlated with poor clinical outcomes. *in vitro* and *in vivo* studies in HCC cell lines corroborated the effect of miR-526b on tumor growth and metastasis. Thus, we suggest that miR-526b loss functions as a pro-cancer factor possibly via SIRT7-mediated ERK pathway in HCC.

## MATERIALS AND METHODS

### Clinical samples

Clinical samples (80 HCC tissues and pair-matched adjacent normal liver tissues) were obtained from HCC patients who had not undergone radiofrequency ablation or chemoembolization in the First Affiliated Hospital of Xi'an Jiaotong University. Samples were pathologically confirmed and rapidly put into liquid nitrogen and 10% formalin after surgical operation. Informed consent was signed by each patient before clinical specimens being collected and used. Details of the clinicopathological data are shown in Table 1. The protocols involved in clinical specimens in this study were permitted by the Research Ethics Committee of Xi'an Jiaotong University.

### Cell culture and transfection

Human HCC cell lines including Hep3B, Huh7, SMMC-7721 and Huh7, and the human immortalized normal hepatocyte cell line (LO2) (Shanghai Institute of Biochemistry and Cell Biology, Chinese Academy of Sciences, Shanghai, China) cultured under standard conditions. Hsa-miR-526b mimics, inhibitors and their control fragments (NC) were produced by GeneCopoeia (Guangzhou, China). SIRT7 expression plasmid (pcDNA3.1-SIRT7) was designed and synthesized by GenePharma (Shanghai, China). All vectors were then transfected into HCC cells with Lipofectamine 2000 (Invitrogen, Carlsbad, CA, USA) following manufactures’ protocols.

### Immunohistochemistry (IHC)

The paraffin sections from HCC tissues were dewaxed, dehydrated, and rehydrated. Then, citrate buffer was used for retrieve antigen, and hydrogen peroxide (3.0%) was used for blocking the endogenous peroxidase activity. After being blocked by 10% goat plasma, SIRT7 primary antibody (sc-365344; Santa Cruz Biotechnology, Santa Cruz, CA, USA) was added to the sections and incubated at 4°C overnight. The biotinylated secondary antibody (ZSGB-BIO, Beijing, China) was applied for detecting the primary antibodies. Counterstained was performed using hematoxylin. DAB solution was carried out for coloration. Cells in five randomly selected high power fields (400× magnification) were calculated for the average of positive rates (0-100%). IHC score was graded as 0, less than 10 %; 1, 10–30 %; 2, 31–50 %; 3, more than 50 %[32]. IHC score ≥ 1 was considered as positive expression of SIRT7.

### Quantitative real-time polymerase chain reaction (qRT-PCR)

RNA was extracted and prepared for qRT-PCR as previously described [33]. Total RNA was reverse-transcribed to cDNA with PrimeScript Reverse Transcriptase kit (Takara, Dalian, China) according to the manufacturer's protocols. By using SYBR Green chemistry, qRT-PCR was implemented with the ABI 7900HT sequence detection machine (Bio-Rad, CA, USA). The target and reference genes (U6 and GAPDH) were amplified in separate wells in triplicate. Gene expressions were calculated with the comparative threshold cycle (2^−ΔΔCT^) approach. The primers used for miR-526b, U6, SIRT7 and GAPDH were synthesized and purchased from Sangon Biotech (Shanghai, China).

### Cell counting Kit-8 (CCK-8) proliferation assay

The HCC cells were seeded onto 12-well plates with 5×10^3^ cells/well, cultured for 24 hours, and transfected with the indicated vectors. Cell Counting Kit-8 (CCK-8; Beyotime, Shanghai, China) assay was performed for detecting cell proliferation. At each day, plates were incubated with CCK8 solution for 2 hours at 37°C. The absorbance rates were measured by VICTOR3™ Multilabel Plate Readers (PerkinElmer Inc., Foster City, CA, USA) at 490 nm.

### Migration and invasion assay

Transwell chambers (coring costar, Cambridge, MA, USA) were employed to evaluate the migratory and invasive abilities of HCC cells. HCC cells were resuspended in serum free DMEM medium and subsequently seeded in the upper chambers. To induce the migration and invasion of HCC cells, the lower chambers were filled with 600μL DMEM supplemented with 20% FBS. 48 hours after cell seeding, HCC cells that migrated or invaded through the membranes (the membranes were covered with 70 μL matrigel) were stained with crystal violet for cell counting under the microscope.

### Western blotting

Total cell lysates were prepared in a 1×sodium dodecyl sulfate buffer and quantified with a BCA protein assay kit (Pierce, Bonn, Germany). Identical quantities of proteins were separated by sodium dodecyl sulfate-polyacrylamide gel electrophoresis and transferred onto PVDF membranes (Bio-Rad, CA, USA). After incubation with primary antibody for overnight, the blots were incubated with secondary antibody (#7074 and #7076; Cell Signaling Technology, Beverly, MA, USA) and detected using a chemiluminescent detection system (Bio-Rad). GAPDH (sc-293335; Santa Cruz Biotechnology, Santa Cruz, CA, USA) was used as a loading control for western blots. SIRT7 (sc-365344), MMP1 (sc-137044) and ERK (sc-514302) antibodies were purchased from Santa Cruz Biotechnology. p-ERK (#4060), c-Myc (#5605), c-Jun (#9165), Cyclin D1(#2978), SNAIL (#3879), HIF-1α (#79233), Ku80 (#2180) and SLUG (#9585) antibodies were obtained from Cell Signaling Technology. The Bio-Rad Gel imaging system (Bio-Rad, Hercules, CA, USA) was used to quantify western blotting data.

### Experimental mouse model

BALB/c nude mice aged 4 week old were subjected to subcutaneous tumor formation and pulmonary metastasis model. SMMC-7721 cells that were transfected with miR-526b mimic and NC mimic, respectively, were subcutaneously injected into the flank of nude mice for 3 weeks or intravenously injected through the tail vein of nude mice and cultivated for 9 weeks. After euthanasia, the lungs were harvested and fixed, paraffin-embedded, sectioned and stained for hematoxylin-eosin (H&E) [34], and the metastatic nodules were counted. All animal experiments were approved by the Ethics Committee of Xi'an Jiaotong University.

### Dual-Luciferase reporter assay

The sequences of SIRT7-3′UTR were cloned into the pmiR-RB-Report™ vector (RIBOBIO, Guangzhou, China), and its corresponding mutant (mt) 3′UTR sequences were subsequently generated using overlap extension PCR and cloned into the pmiR-RB-Report™ vector. Pmir-RB-SIRT7 or pmir-RB-SIRT7-mt was transfected into Hep3B cells with corresponding miRNA vectors by lipofectamine-mediated gene transfer. The relative luciferase activity was normalized to Renilla luciferase activity 48h after transfection.

### Statistical analysis

Data were presented as Mean ± SD and analyzed by GraphPad Prism 5 software (GraphPad Software, Inc, San Diego, CA, USA) and the SPSS statistical package for Windows Version 17.0 (SPSS, Chicago, IL, USA). Chi-squared test, multivariate Cox's analysis, Student's t-test, ANOVA, Kaplan-Meier method, Log-rank test and Pearson's correlation analysis were performed for statistical analysis. A *P*-value < 0.05 was considered statistically significant. ^*^P<0.05.

## SUPPLEMENTARY MATERIALS TABLE AND FIGURE



## Abbreviations

HCC: hepatocellular carcinoma
TNM: tumor-node-metastasis
SIRT7: sirtuin 7
EMT: epithelial-to-mesenchymal transition
ESCC: esophageal squamous cell carcinoma
NSCLC: non-small cell lung cancer
MMP1: matrix metalloproteinase 1
HIF-1α: hypoxia-inducible factor 1-alpha
IHC: immunohistochemistry
qRT-PCR: quantitative real-time polymerase chain reaction
CCK-8: Cell Counting Kit-8
